The article "Analysis and Research on Human Movement in Sports Scene" was published in 2021. Journal: Comput Intell Neurosci.

# Analysis and Research on Human Movement in Sports Scene

**DOI:** 10.1155/2021/2376601

**Published:** 2021-12-23

**Authors:** Yan Wang, Yuchen Zhang, LinJun Shen, ShuMing Wang

**Affiliations:** ^1^Institute of Physical Education of Chaohu University, Chaohu 238240, China; ^2^School of Physical Education and Health, East China Normal University, Shanghai 200241, China; ^3^Shenyang Agricultural University College of Forestry, Shenyang 110866, China

## Abstract

As a whole-body sport, skipping rope plays an increasingly important role in daily life. In rope-skipping education, due to the lack of professional teachers, the training efficiency of students is low. The rope-skipping monitoring device is heavy and expensive, and the cost of labor statistics and energy consumption are high. In order to quickly analyze the movement process of students and provide correct guidance, this article implements the movement analysis method of the human body movement process. The problem of limb posture analysis in rope skipping is transformed into a multilabel classification problem, a real-time human motion analysis method based on mobile vision is proposed, and the algorithm model is verified in the rope-skipping scene. The experimental results prove that this paper proposes the improved algorithm, which achieved the expected effect. In the analysis of rope-skipping action, the choice of hyperparameters during the experiment is introduced, and it is verified that the proposed ALSTM-LSTM can solve the problem of multilabel classification in the rope-skipping process. The accuracy rate reaches 95.1%, and it can provide the best in all indicators and good performance. It is of great significance for movement analysis and movement quality evaluation during exercise.

## 1. Introduction

In the study of human motion recognition, we apply a convolution neural network to it, choose a one-dimensional CNN + LSTM algorithm as the optimal algorithm, and then select sensors that can support smart wearable devices, build a recognition network model, and then process the collected data. This method can be used under any circumstances, and the cost is relatively low, which is mostly used in sports events [1]. At present, Bluetooth is widely used in wireless technology. In order to evaluate the performance of Bluetooth, especially the body area network (BAN) using magnetic inertial sensor units (M-IMUs) for human motion tracking, we propose a method for throughput performance in general sensor network applications [2]. The analysis of human motion is of great significance in the diagnosis of musculoskeletal diseases. Usually, we use micro-Doppler features measured by the radar to analyze human motion, but deep learning requires a huge amount of data and the cost is quite high. Therefore, we have studied a more accurate method to improve the analysis, that is, to expand the mode of micro-Doppler data of human motion by generating countermeasure networks (GANs) [3]. Detection of human presence in video streams is a challenging research. Therefore, we propose a method to analyze human motion in the dark by using a digital image processing technology, which can mainly model, analyze, and identify human motion in walking and running in video stream [4].

The article "Analysis and Research on Human Movement in Sports Scene" was published in 2021. Journal: Comput Intell Neurosci.

In recent years, with the continuous development and application of computer technology and artificial intelligence technology, human motion analysis technology based on vision has been rapidly developed and highly valued [5, 6]. Human motion analysis based on vision is also a challenging subject in computer vision, mainly involves model recognition, image processing, virtual reality, and other disciplines, and has a wide application prospect in the field of human-machine interaction. The core problem of motion analysis is the inference of human body shape, which is an important research topic in the field of computer vision. Artificial intelligence technology has penetrated into sports training projects, and many intelligent hardware and software have been produced in sports training. The continuous penetration of artificial intelligence technology in sports training has promoted the development of sports. Sight, hearing, art, hand, foot, wrist, and shoulder movements require rhythmic coordination. It has moderate overall strength, physical strength, ability, and coordination, especially suitable for physical education in primary and secondary schools. There is a serious shortage of professional physical education teachers in compulsory education in China. According to the statistics of the Ministry of Education, the proportion of professional physical education teachers in compulsory education in China is 300,000 at present. The growth of qualified PE teachers needs the accumulation of professional learning and long-term educational experience, which further aggravates the seriousness of the lack of professional PE teachers' skills. Schools cannot keep track of each student's learning and training progress, and it is difficult to educate different people for the second time. The traditional control equipment for skipping rope in college entrance examination is bulky and expensive, and the cost and labor energy consumption are too high. The key to improve the performance of suspension test is to automatically and quickly analyze whether the suspension action conforms to the standard and to provide correct driving and training plans, so as to better apply the action analysis of suspension test to skipping rope training in complex situations. In view of the above problems, this paper mainly combines deep learning and multilabel action analysis [7], and a new algorithm for analyzing artistic movements in the process of multilabel skipping rope is designed. It is suitable for the analysis of skipping rope and jumping action of two legs in the entrance examination of middle school [8]. It is suitable for complex indoor and outdoor environment and does not need to master any special equipment. Compared with the traditional complex design, it can effectively improve the detection accuracy and reduce the false alarm rate and alarm system, thus effectively solving the real-time analysis problem and accurate analysis, and improving the grades of middle school students. The application of deep learning model in motion prediction can deeply analyze and predict motion rules and can effectively determine the corresponding motion rules and trajectories. By mastering the planning of sports, the efficiency and standardization of sports can be effectively improved.

The article "Analysis and Research on Human Movement in Sports Scene" was published in 2021. Journal: Comput Intell Neurosci.

## 2. Introduction of Related Technologies

### 2.1. Deep Learning Method

The purpose of deep learning model design is to extract low-dimensional features of data and transform them into high-dimensional features. Deep learning is different from traditional machine learning algorithms and needs a lot of data support. The larger the amount of data, the more knowledge the model learns, and the better the effect. With the advent of 5G era, the generation of large-capacity data provides data support for deep learning mode. At the same time, the development of software and hardware equipment also applies the deep learning mode to the actual environment [9, 10].

#### 2.1.1. Cyclic Neural Network Model

Cyclic neural network (RNN) is one of the most widely used basic structures in deep learning. Different from general feedforward neural networks, cyclic neural networks allow a transverse connection of some neural units. In the cyclic neural network, the input data of the current layer and the output data of the previous layer need to be combined into the current layer, and the data can be updated through the cyclic calculation of the first layer, so the cyclic neural network has a certain storage function for the data of the previous layer. Because the cyclic neural network has a certain storage capacity, it can capture the information in data and learn the logical relationship between the data before and after, so RNN is often used to solve the problem of time series characteristics in data. In order to detect and identify track circuit faults in time, an LSTM structure network is used to learn the temporal and spatial correlation of circuit signal data. In order to solve the problem that is difficult to detect images at the end of restoration and diastole in ultrasonic heartbeat images, Dezak et al. use an RNN structure to process them and consider the time dependence between frames. A deep learning model including an RNN structure of Lee et al. is used for human motion recognition [11, 12]. We propose an RNN model, such as Zhang, which realizes character emotion recognition by processing EEG and facial expression image data [13]. Zollavari and others put forward a model based on the RNN system structure, which is used to detect the running state of the transformer and evaluate the mechanical integrity of the transformer. Zhang and others put forward the framework of Chinese character recognition model and Chinese character generation model based on the RNN method [14]. Ma et al. proposed a method based on LST, which can effectively extract the state information of broadcast channel and the characteristics of RF equipment to identify illegal broadcast signals. Kim et al. use the RNN structure for disease prediction. Cyclic neural networks are very sensitive to the temporal characteristics of sequential data, and models based on the RNN structure can be given priority [15].

The article "Analysis and Research on Human Movement in Sports Scene" was published in 2021. Journal: Comput Intell Neurosci.

The structure of the cyclic neural network is shown in Figure 1. A is the parameter between the input layer and the hidden layer, B is the parameter between the hidden layer and the hidden layer, and C is the parameter between the hidden layer and the output layer. RNN is a deep neural network, but the parameter layer is shared, so there are only three weight matrices: A, B, and C. This parameter sharing structure has two advantages: (1) the length of input and output of the learning model is the same, regardless of the length of the sequence; (2) the parameters of each time step are the same, so the same transfer function can be used for learning. Cyclic neural networks have serious disadvantages; that is to say, it is difficult to learn long-term dependence. As shown in Figure 2, black circles are used to represent key information. As the network executes backward step by step, the current important information is constantly “diluted,” and the first information is almost useless in the seventh cycle. This is the reason why it is difficult for cyclic neural networks to learn long-term dependence [16].

The long-term storage network is based on the improved variant of the abovementioned cyclic neural network, which optimizes the long-term dependency difficulty and gradient disappearance problems caused by the long learning period in the common cyclic neural network. The LSTM includes storage cells, input gates, output gates, and forgetting gates. Figure 2 is a schematic diagram of the structure of a single-cell LSTM. The input gate, output gate, and forgetting gate are three sigmoid neurons, and their output is “0” or “1,” which means “off” or “on” of a certain function. Similar to RNN, the input is the integration of the input at the current moment with the hidden layer output at the previous moment. However, LSTM in one direction can only get results from one direction when processing sequence data. To solve this problem, Gravies et al. proposed a bidirectional long-time storage network (Bi-SLSTM) composed of forward LSTM and reverse LSTM, which can effectively retrieve bidirectional meaning information of sequence data [17, 18].

The article "Analysis and Research on Human Movement in Sports Scene" was published in 2021. Journal: Comput Intell Neurosci.

### 2.2. 2D Human Pose Estimation Based on OpenPose

#### 2.2.1. OpenPose Network Architecture

As shown in Figure 3, the OpenPose network structure includes upper and lower parts of the whole network. The previous network is used to predict the reliability diagram L of skeleton joints, and the next network is used to predict some affinity vector fields S. The two parts can be iterated, respectively, forecast.

First a front feature of an input image is extracted in the vgg-19 described previously and a set of feature maps *f* are output. Then, the OpenPose network generates a set of confidence graphs and some affinity vector fields, which are *S*^*l*^ = *ρ*^*l*^(*F*) and *L*^*l*^ = Ø^*l*^(*F*), respectively, where *ρ*^*l*^(*F*) and Ø^*l*^(*F*) are inferred from the first feature extraction of vgg-19, and each part can be iterated separately. In the iterative process, the output of the result inferred from the previous feature extraction and the feature map F of the original image are used as inputs to the current network of each part to produce a more accurate prediction result. Formulas (1) and (2) show the specific process of prediction, where *ρ*^*t*^ and Ø^*t*^ are the results in the middle of step *t* [19, 20].

(1) $$\begin{array}{c} S^{t}=\rho^{t}\left(F,S^{t-1},L^{t-1}\right),\;\forall t\geq 2, \end{array}$$

(2) $$\begin{array}{c} L^{t}=\emptyset^{t}\left(F,S^{t-1},L^{t-1}\right),\;\forall t\geq 2. \end{array}$$

The OpenPose network uses loss functions at the end of the upper and lower parts. Therefore, the result of each part of OpenPose repeated prediction is taken as the loss function of the upper and lower parts, and each loss function is weighted in space by using an L2 loss function between the predicted and actual values. The total loss function of the two parts of the T-stage network is shown in the following formulas:

(3) $$\begin{array}{c} f_{S}^{t}=\overset{J}{\underset{j}{\sum }}\underset{p}{\sum }W\left(p\right)\times S_{j}^{t}\left(p\right)-S_{j}^{*}{\left(p\right)}_{2}^{2}, \end{array}$$

(4) $$\begin{array}{c} f_{L}^{t}=\overset{C}{\underset{c=1}{\sum }}\underset{p}{\sum }W\left(p\right)\times L_{c}^{t}\left(p\right)-L_{c}^{*}{\left(p\right)}_{2}^{2}, \end{array}$$

where *S*_*j*_^*∗*^ represents the position confidence map of the correct label of the image, *L*_*c*_^*∗*^ represents the position affinity vector field of the true label of the image, and W is a binary mask that avoids error penalty in some cases. When P has no label, the OpenPose network still performs prediction, and *W* can avoid error punishment for data without label. The final overall objective function is as follows [21]:

(5) $$\begin{array}{c} f=\overset{T}{\underset{t=1}{\sum }}f_{S}^{t}+f_{L}^{t}. \end{array}$$

The article "Analysis and Research on Human Movement in Sports Scene" was published in 2021. Journal: Comput Intell Neurosci.

## 3. Motion Analysis Algorithm in Rope-Skipping Scene

Motion analysis in motion process based on computer vision is a complex problem, especially in the analysis of violent motion. In order to explain the body movements when shaking your legs and dancing in detail, this chapter introduces the model of building a network using deep learning. This chapter mainly introduces the research content [22].

### 3.1. Definition of the Problem

The content of this study is the realization of an intelligent motion alibi system. It involves data collection and processing, resource extraction, data transmission, and network model design. This paper provides a real-time human motion analysis method based on mobile vision. Through the training of two swinging feet in senior high school entrance examination, the problems of real-time motion analysis and evaluation of EM body motion quality are solved and the general analysis of human motion only pays attention to the overall performance. Specifically, it does not involve all types of body movements, so it cannot operate effectively in complex environments. In order to solve this problem effectively, the operation analysis algorithm designed in this paper is based on the deep learning model. Therefore, in the selection of deep learning model, the network model of CNN structure and LSTM network combination model of attention mechanism are used to obtain robust data through CNN and analyze whether there is a reference for body movement together with the LSTM model.  Figure 4 shows the specific flowchart. From the flowchart, it can be seen that the foot motion analysis mainly includes two modules: one module is used to obtain key information from human body, and the other module is used to mathematically model the obtained key information and establish a multilabel classification network model [23].

The article "Analysis and Research on Human Movement in Sports Scene" was published in 2021. Journal: Comput Intell Neurosci.

At the end of analyzing the body movements of athletes in the process of jumping their legs, first, the video stream data are transformed into key human body coordinate data by the improved open network model, the time series of key coordinates of human body is established, and the data are preprocessed. The coordinates of main points in the process of robust skipping rope are obtained because the key coordinates of the main form are time series. There is a certain relationship between them. This paper also applies the LSTM model to submit behavior analysis by transforming the algorithm into a multi-label classification algorithm. The posture analysis problem in the process of rope skipping can evaluate whether athletes have action benchmarks in the process of rope skipping. The content of this study is to analyze the one-minute jumping posture of both feet in the entrance examination of middle school. The after-sales analysis of rope can be divided into whether the body stands or not. Are your left arm and body tight? Whether the right arm and body are tight. Is the left arm symmetrical with the right arm? Does your left arm bounce? Skipping rope with your right arm? These body movements are selected by professional PE teachers by checking the average input. The problem is defined as a preprocessor in a given string group skipping record and record sequence data group. A reliable data sequence *D* = (*r*_1_, *r*_2,_…, *r*_*m*_) is obtained, where *r*_*j*_, *i* = 1,…, and *m* represents *m* sequences of data; the tag set *L* = {*l*_1_,…, *l*_*n*_},*l*_*j*_, where *j* = 1,…, *n* represents the tag of the member when rope skipping. Each MS D record is associated with a plurality of MS L tags. The analysis of multitagged gestures can be expressed by tuples (*r*_*i*_, *Y*_*i*_), in which *Y*_*i*_ ∈ *L* our goal is to design and implement a tag classification model, which can judge the limb tags *Y*_*i*_′ during skipping rope according to the new posture data set*r*_*i*_′.

### 3.2. Network Framework Design

#### 3.2.1. MobileNetv2 Framework

A MobileNetv2 network was proposed by Google team in 2018. The point in MobileNetv2 is the defect structure, as shown in Figure 5.  Figure 5(a) is the residual structure of ResNet network, and Figure 5(b) is the deflation structure of MobileNetv2. When the magnetoresistive activation function is used, the information of higher order elements is lost less, so the low-size information is usually lost when the magnetoresistive activation function is used. Therefore, in the final stage, a linear activation function is used to keep the low-dimensional information resources in a 1 convolution layer [24].

The article "Analysis and Research on Human Movement in Sports Scene" was published in 2021. Journal: Comput Intell Neurosci.

Table 1 shows the structure of the MobileNetv2 network. *T* denotes the expansion factor, C denotes the channel of the feature output matrix, *N* denotes the number of repetitions of the reverse residual structure, and *S* denotes the step distance.  Figure 6 shows a network structure with asynchronous long intervals.

#### 3.2.2. ALSTM-LSTM Network Framework

In this paper, the position analysis of human body in rope skipping is transformed into a multilabel problem based on the time ratio. LSTM plays an important role in processing and global storage. In order to maintain the performance of BOM in time series, attention mechanism is also a global processing method. It can apply attention mechanism to LSTM to improve the performance of LSTM, which is equivalent to significantly increasing the overall information modeling process of LSTM. FIM can compensate for what LSTM did not learn and failed. Therefore, inspired by LSTM mechanism and attention, this paper proposes a method to apply LSTM focusing mechanism and classify multiple tags in combination with a single LSTM.  Figure 7 shows the ALSTM-LSTM network framework.

ALSTM-LSTM consists of five layers: entry layer, batch normalization layer, ALSTM-LSTM layer, binding layer, and sigmoid layer.  Figure 8 shows the detailed parameters of the ALSTM-LSTM system structure.

This article adds a buffer layer before using LSTM and ALSTM layers. In addition, the ALSTM-LSTM model defines the activation function as the S-shaped activation function of the last layer and selects the binary transverse entropy loss function as the loss function because the multilabel classification problem is discussed according to the transformation method of multilabel algorithm.

### 3.3. Optimal Attitude Estimation Algorithm

Among the two branches of OpenPose, one branch is used to predict the confidence maps (S) of key points, that is, the probability values of key points, and the other branch is used to predict the PAFS(L) affinity domain between two key points. Losses at different stages represent the L2 tree between the expected values and the actual values (*S*^*∗*^, *L*^*∗*^) of S and I, and w(P) is 0 or 1. When it is 0, it means that the key point is missing, and the loss is not calculated. The loss of different stages is calculated as follows:

(6) $$\begin{array}{c} f_{S}^{t}=\overset{J}{\underset{j}{\sum }}\underset{p}{\sum }W\left(p\right)\cdot S_{j}^{t}\left(p\right)-S_{j}^{*}{\left(p\right)}_{2}^{2},\\ f_{L}^{t}=\overset{C}{\underset{c=1}{\sum }}\underset{p}{\sum }W\left(p\right)\cdot L_{c}^{t}\left(p\right)-L_{c}^{*}{\left(p\right)}_{2}^{2}. \end{array}$$

The total loss is based on the sum of the losses at each stage.

(7) $$\begin{array}{c} f=\sum_{t=1}^{T}f_{S}^{t}+f_{L}^{t}. \end{array}$$

In order to further improve the generalization ability and accuracy of the attitude estimation algorithm, FIM introduces two weights and a penalty term in the total loss function: *f*=∑_*t*=1_^*T*^(*αf*_*s*_^*t*^+*βf*_*L*_^*t*^+*θ*). By introducing weights, the influence of losses in two branches on the results is analyzed.

The article "Analysis and Research on Human Movement in Sports Scene" was published in 2021. Journal: Comput Intell Neurosci.

## 4. Experiment and Analysis

A two-stage network model is established to analyze the movement of legs in the central entrance examination. The first stage is USADA, which is used to obtain the key coordinates of human body. In the second stage, this chapter introduces two necessary data in the experimental process, introduces the collection and preprocessing process of skipping data set in detail, and makes experimental comparison and analysis.

### 4.1. Introduction to Data Sets

#### 4.1.1. MPII Data Set

The MPII data set contains many photos of everyday life. There are 24,920 photos, 40,522 human samples, 3,844 training groups, and 1,758 test groups in this data set. The method proposed by Tompson et al. was used in the experiment. The number of training groups was 25863, verification groups were 2958, and test groups were 11701. MPII data set shows 16 kinds of human joints and the total of 15 key coordinates output by a thermal diagram. MPII data sets are challenging, including more samples with complex background, severe occlusion, and poor lighting conditions [25].

#### 4.1.2. Rope-Skipping Data Set

The data set of this study comes from an experimental middle school. The skipping video data collected by the institute were taken in different scenes by mobile phones and start from the front. The video is recorded in an MP4 format. Different portable devices have different image pixels. Now, 200 high school students collect data from a one-minute skipping video. Among them, there are 96 boys, 104 girls, and 52 girls. 80 people graduated from high school in two years, and 68 people graduated from high school in three years. Students are between 11 and 15 years old.  Figure 9 shows the distribution histogram of men and women in Series 3.

Data labels are marked in a chronological order by professionals who analyze images. The data labels are SEIS markers, which define the left and right arms as constrained horizontally, body upright (body straight, but not hard), left arm and strong body, right arm and strong body, left wrist swing rope, right arm swing, and right arm swing. The choice of these labels is defined according to the technology of skipping rope in the entrance examination. Please refer to Table 2 for details. The *X* feature set and Y tag set of the constructed data represent a DX-dimensional D-dimensional input space = *R*, the size of *D* is 36, *Y* = {0,1}^*q*^ is the tag space of possible tags, the size of *q* is 6, *T*=(*x*^*i*^, *y*^*i*^)*|*1 ≤ *i* ≤ *m*, where *m* represents the size of the data set, *x*^*i*^ ∈ X is a 36-dimensional vector, and *y*^*i*^ ∈ Y is a tag subset of Y.

The article "Analysis and Research on Human Movement in Sports Scene" was published in 2021. Journal: Comput Intell Neurosci.

### 4.2. Evaluation Indicators

#### 4.2.1. Evaluation Index of Human Key Point Detection

Frequently used evaluation indexes of human skeleton points include ok *s*, average accuracy of AP and mAP. The purpose of oks is to calculate the actual value and predict the similarity of important parts of human body. The calculation method is

(8) $$\begin{array}{c} OKS_{p}=\frac{\sum_{i}\exp\left\{-\left(d_{pi}^{2}/2S_{p}^{2}\sigma_{i}^{2}\right)\right\}\sigma \left(v_{pi}>0\right)}{\sum_{i}\sigma \left(v_{pi}>0\right)}. \end{array}$$

The AP index is used to calculate the accuracy percentage of test set, and the calculation methods of single-person pose estimation and multiperson pose estimation are different.

(9) $$\begin{array}{c} AP_{\text{double}}=\frac{\sum_{m}\sum_{p}\delta \left(oks_{p}>T\right)}{\sum_{m}\sum_{p}1},\\ AP_{\text{single}}={\hat{\rho }}_{k}=\frac{{\hat{\gamma }}_{k}}{{\hat{\gamma }}_{0}}=\frac{cov\left(X_{t},X_{t-k}\right)}{\sigma_{X_{t}},\sigma_{X_{t-k}}}=\frac{\sum_{i=1}^{n=k}\left(X_{t}-\bar{X}\right)\left(X_{t-k}-\bar{X}\right)}{{\sum_{i=1}^{n=k}\left(X_{t}-\bar{X}\right)}^{2}}. \end{array}$$

MAPs refer to setting different values for artificial threshold *T* in AP indicators, then obtaining multiple AP indicators, averaging multiple AP indicators, and finally obtaining MAP.

#### 4.2.2. Evaluation Index of Multilabel Classification

Evaluation indexes based on multilabel classification usually include Accuracy, F1-Score, Preference, and Recall. Accuracy means that the number of logarithmic samples of the classifier in the test set accounts for the percentage of all samples in the classification process.

(10) $$\begin{array}{c} \text{Accuracy}=\frac{\sum_{i=1}^{l}\left(TP_{i}+TN_{i}/TP_{i}+FP_{i}+TN_{i}+FN_{i}\right)}{l}. \end{array}$$

F-Score is the product of weighting Preference and Recall. Accuracy refers to the proportion of accurately predicted samples to positive samples in the test set, and the Recall rate refers to the proportion of accurately predicted positive samples to positive samples.

(11) $$\begin{array}{c} \text{Precision}=\sum_{i=1}^{l}k_{i}\left(\frac{TP_{i}}{TP_{i}+FP_{i}}\right),\\ \text{Recall}=\sum_{i=1}^{l}k_{i}\left(\frac{TP_{i}}{TP_{i}+FN_{i}}\right),\\ F1=\sum_{i=1}^{l}k_{i}\left(\frac{2Precision_{i}Recall_{i}}{Precision_{i}+Recall_{i}}\right). \end{array}$$

The article "Analysis and Research on Human Movement in Sports Scene" was published in 2021. Journal: Comput Intell Neurosci.

### 4.3. Analysis of Experimental Results

#### 4.3.1. Experimental Environment Setting

The development of deep learning mode needs open source frameworks such as TensorFlow, Keras, Caffe, and PyTorch. They need to use the professional language for programming experiments. A deep learning mode needs a lot of computer resources in the training process and also has certain requirements for computer equipment:

1. The software environment is the process of gesture estimation and skipping motion analysis, and the codes are all made in PyCharm and Jupyter Notebook. Here, PyCharm is a python language development tool, with powerful functions. Jupyter Notebook is an interactive application of web programming, and the results of each step can be easily seen on the Jupyter Notebook. It is very convenient to adjust in the training of deep learning mode. In addition, the Jupyter Notebook can analyze the data and visualize it.
2. The hardware environment of this experiment is as follows: CPU is Intel Commie 7-8700K, 3.70 GHz, and 32G memory. GPU is GTX1080TI.

#### 4.3.2. Experimental Analysis of Attitude Estimation Results

In order to improve the accuracy and efficiency of pose estimation, the feature extraction model vgg-19 in the initial stage of OpenPose is replaced by the lightweight network model MobileNetV2, and the quota and penalty items are introduced into the final loss function. Although the accuracy is not expected to be improved by using MobileNetV2 in the local experimental platform, the overall parameters of the model are reduced.  Table 3 shows the results on the MPII data set. The results show that the improved model structure can meet the experimental requirements of this paper.

#### 4.3.3. Analysis of Experimental Results of Multilabel Classification of Skipping Movements

When analyzing skipping operation, this paper first uses a single-layer LSTM structure to compare the influence of superparameter selection results in LSTM. Unity in LSTM is set to 32, 64, 128, and 256, respectively. Unity refers to the number of neurons in the hidden layer of each LSTM unit, and the batch sizes are set to 16, 32, 48, 64, 80, 100, 128, 150, 200, and 256, respectively. The optimum performance is 0.896 when the batch-processing size is 100 in the number of units (64) of LSTM.

Figure 10 shows the ROC and AUC curves in a single-layer LSTM when the hidden unit is 64 and the batch size is 100, and the accuracy of each label is 0.785, 0.843, 0.907, 0.768, 0.838, and 0.953, respectively.

Rope skipping motion analysis process is actually a long sequence analysis process, and we need to use a sliding window to segment the data. Among them, in order to find the proper sliding window length, 10 frames of cumulative coordinates and 15 frames of cumulative coordinates are needed, respectively, three groups of 20 frames of cumulative coordinates are needed, and the step is set as an experiment of 30% data superposition.  Figure 11 shows LSTM performance at 64, batch size at 100, and sliding window lengths at 10, 15, and 20. Experimental results show that the performance of LSTM is the best when the length of the sliding window is 15.

The article "Analysis and Research on Human Movement in Sports Scene" was published in 2021. Journal: Comput Intell Neurosci.

To further verify the effectiveness of the model proposed in this paper, we set the number of hidden units in ALSTM-LSTM to 64. When the size of batch processing reaches 100 and the length of a sliding window is 15, it can be seen from Figure 12 that the accuracy of each label is improved compared with the single-layer LSTM model.

The ALSTM-LSTM model was compared with several models to further validate its performance, as shown in Table 4. As a result, in the multilabel classification problem of skipping operation analysis, the deep learning model is superior to the traditional machine learning algorithm. This paper further verifies the influence of batch normalization method on the model performance. In the last skipping operation analysis of the experiment, the structure of the ALSTM-LSTM system provides the highest performance in all indicators, indicating that the performance of SVM is the worst.

## 5. Conclusion

In order to solve the difficult problem of skipping motion analysis, this paper studies the motion analysis under the motion scene. First, a deep learning framework is proposed to obtain the coordinates of key points. The coordinates are optimized to obtain the sequence of key points of human body. The problem of judging whether the obtained key point sequence is standard is transformed into a multilabel classification problem, and a multilabel classification model ALSTM-LSTM is proposed to classify labels, which finally achieves 95.1% accuracy and achieves the best in all indexes, which is of great significance for motion analysis and motion quality evaluation in the process of motion. Through the classification of human movement rules, this paper puts forward a human motion model based on mobile vision, which can effectively improve the efficiency of motion. The main work in the future is to analyze the influence of the correctness of motion posture on health and find out a kind of exercise mode, which is suitable for high efficiency and health from a large number of exercise data sets.

## Figures and Tables

**Figure 1:** Schematic diagram of cyclic neural network development.

The article "Analysis and Research on Human Movement in Sports Scene" was published in 2021. Journal: Comput Intell Neurosci.

**Figure 2:** Schematic diagram of long-term dependence difficulty of the cyclic neural network.

**Figure 3:** OpenPose network structure diagram.

**Figure 4:** Design flowchart of the skipping action analysis model.

**Figure 5:** (a) Residual block. (b) Inverted residual block.

**Figure 6:** Different network architectures of Stride. (a) Stride = 1 block. (b) Stride = 2 blocks.

**Figure 7:** ALSTM-LSTM network frame diagram.

**Figure 8:** ALSTM-LSTM structure diagram.

**Figure 9:** Rope-skipping data set distribution histogram.

**Figure 10:** ROC and AUC curves in a single-layer LSTM.

**Figure 11:** Selection of the sliding window.

**Figure 12:** ROC and AUC curves of ALSTM-LSTM.

**Table 1:** MobileNetv2 network structure.

Input	Operator	*t*	*c*	*n*	*s*
224^2^ × 3	Conv2d	—	32	1	2
112^2^ × 32	Bottleneck	1	16	1	1
112^2^ × 16	Bottleneck	6	24	2	2
56^2^ × 24	Bottleneck	6	32	3	2
28^2^ × 32	Bottleneck	6	64	4	2
14^2^ × 64	Bottleneck	6	96	3	1
14^2^ × 96	Bottleneck	6	160	3	2
7^2^ × 160	Bottleneck	6	320	1	1
7^2^ × 320	Con2d 1 × 1	-	1280	1	1
7^2^ × 1280	Avgpool 7 × 7	-	-	1	-
1 × 1 × 1280	Con2d 1 × 1	-	k	-	

**Table 2:** Names of limb movement markers.

Classification	Description
Keep your body upright	Judge whether the whole-body remains straight but not stiff
The left big arm and the body tighten up	Judge whether the left big arm is next to the trunk of the body
The right big arm and the body tighten up	Judge whether the right big arm is next to the trunk of the body
Left wrist rocking rope	Determine if it is the wrist that drives the rope to rotate
Right wrist rocking rope	Determine if it is the wrist that drives the rope to rotate
Keep your left and right arms level	Judge whether the left arm is symmetrical with the right arm

**Table 3:** Experimental results on MPII data sets.

Method	Head	Shoulder	Elbow	Ability	Hip	Knee	Ankle	mAP
Deepcut	78.4	72.5	60.2	51.0	57.2	52.0	45.4	59.5
OpenPose	91.2	87.6	77.7	66.8	75.4	68.9	61.7	75.6
The improved method in this paper	93.3	88.1	75.6	72.2	78.3	70.0	60.8	76.9

**Table 4:** Comparison of the ALSTM-LSTM model with other models.

Model	Accuracy (%)	Precision (%)	Recall (%)	F1 (%)
ALSTM-LSTM	95.1	95.6	94.1	94.8
ALSTM-BN	92.8	94.5	89.6	91.9
LSTM-BN	92.7	93.0	91.2	92.1
ALSTM	91.2	91.9	88.9	90.3
LSTM	89.6	88.8	89.2	88.7
ML-KNN	79.6	75.3	74.8	74.4
SVM	76.7	74.2	76.6	76.3

## Data Availability

The experimental data used to support the findings of this study are available from the corresponding author upon request.
